# MicroRNA-489 Promotes the Apoptosis of Cardiac Muscle Cells in Myocardial Ischemia-Reperfusion Based on Smart Healthcare

**DOI:** 10.1155/2022/2538769

**Published:** 2022-01-07

**Authors:** Wenhua Li, Yixin Zhang, Jian Wang, Qiang Li, Di Zhao, Bozan Tang, Shiwei Wang, Haifeng Shao

**Affiliations:** ^1^Department of Cardiovascular Medicine, The Third Affiliated Hospital of Qiqihar Medical University, Qiqihar 161000, China; ^2^Department of Endocrinology, The Second Affiliated Hospital of Qiqihar Medical University, Qiqihar 161000, China; ^3^Department of Medical Services, The Third Affiliated Hospital of Qiqihar Medical University, Qiqihar 161000, China

## Abstract

With the development of information technology, the concept of smart healthcare has gradually come to the fore. Smart healthcare uses a new generation of information technologies, such as the Internet of Things (loT), big data, cloud computing, and artificial intelligence, to transform the traditional medical system in an all-around way, making healthcare more efficient, more convenient, and more personalized. miRNAs can regulate the proliferation, differentiation, and apoptosis of human cells. Relevant studies have also shown that miRNAs may play a key role in the occurrence and development of myocardial ischemia-reperfusion injury (MIRI). This study aims to explore the effects of miR-489 in MIRI. In this study, miR-489 expression in a myocardial ischemia-reperfusion animal model and H9C2 cells induced by H/R was detected by qRT-PCR. The release of lactate dehydrogenase (LDH) and the activity of creatine kinase (CK) was detected after miR-489 knockdown in H9C2 cells induced by H/R. The apoptosis of H9C2 cells and animal models were determined by ELISA. The relationship between miR-489 and SPIN1 was verified by a double fluorescence reporter enzyme assay. The expression of the PI3K/AKT pathway-related proteins was detected by Western blot. Experimental results showed that miR-489 was highly expressed in cardiac muscle cells of the animal model and in H9C2 cells induced by H/R of the myocardial infarction group, which was positively associated with the apoptosis of cardiac muscle cells with ischemia-reperfusion. miR-489 knockdown can reduce the apoptosis of cardiac muscle cells caused by ischemia-reperfusion. In downstream targeting studies, it was found that miR-489 promotes the apoptosis of cardiac muscle cells after ischemia-reperfusion by targeting the inhibition of the SPIN1-mediated PI3K/AKT pathway. In conclusion, high expression of miR-489 is associated with increased apoptosis of cardiac muscle cells after ischemia-reperfusion, which can promote the apoptosis after ischemia-reperfusion by targeting the inhibition of the SPIN1-mediated PI3K/AKT pathway. Therefore, miR-489 can be one of the potential therapeutic targets for reducing the apoptosis of cardiac muscle cells after ischemia-reperfusion.

## 1. Introduction

Acute coronary syndrome (ACS) is a group of clinical syndromes caused by acute myocardial ischemia due to coronary thrombosis, with high mortality. Timely restoration of the effective blood flow in cardiac muscles can significantly reduce the cardiac cell injury caused by ischemia and fully improve the prognosis of patients, which is the first-line treatment protocol for ACS [1]. However, restoring blood flow does not necessarily restore the functions of injured cardiac muscle cells and may also lead to reperfusion injury, causing further deterioration of the disease. This tissue injury caused by the recovery of blood flow after ischemia in cardiac muscle cells is called myocardial ischemia-reperfusion injury (MIRI), which may cause irreversible injury to the structure and functions of cardiac muscles, as an important factor affecting the prognosis of patients with ACS. The mechanism of ischemia-reperfusion injury may be a free radical injury, calcium overload, energy metabolism disorder of cardiac muscles, injury to the antioxidant system of endothelial cells, the apoptosis of cardiac muscle cells, and so on [2–4] among which, apoptosis plays a crucial role in the pathogenesis of MIRI, associated with its prognosis. Therefore, it is crucial to clarify the factors affecting the apoptosis of cardiac muscle cells after myocardial ischemia-reperfusion.

MicroRNA (miRNA) is an endogenous noncoding single-chain small RNA molecule consisting of 21–23 bases, which hybridizes with some of the partial nontranslated regions of messenger RNA for target genes, guiding the assembled ribonucleic protein complex to cut mRNA or inhibit its translation. Therefore, microRNA can regulate the expressions of target genes by acting as a posttranscriptional regulator for gene expression. The expression and functions of microRNA are closely related to the occurrence and development of many diseases. In recent years, it has been gradually recognized that microRNA may play a key role in the occurrence and development of MIRI, associated with myocardial autophagy, apoptosis, necrosis, and oxidative stress, inflammation, and mitochondrial dysfunction [5–8]. miR-489 is a microRNA that can regulate the proliferation, differentiation, and apoptosis of human cells, commonly considered an inhibitory factor for oncogenes or tumors [9–11]. Recent relevant literature has shown that it may be crucial in the occurrence and development of ischemia-reperfusion [12, 13]. Its clinical significance, biological functions, and potential mechanism in ischemia-reperfusion are not completely clear. This study aims to explore the effects of miR-489 in MIRI and its specific mechanism to provide a reference for the treatment of MIRI.

## 2. Experimental Methods

### 2.1. Target Prediction

TargetScan database was adopted for querying, and it was found that SPIN1 may be a downstream target for miR-489.

### 2.2. Establishment of Animal Model

SD rats aged 8 to 10 weeks purchased from Shanghai Slaccas Experimental Animal Co., Ltd. (Animal approval number 2015000504404) to establish a myocardial ischemia-reperfusion model were divided into two groups: control group (*n* = 16) and myocardial ischemic-reperfusion group (MI group, *n* = 16). A myocardial infarction model was established by clamping the left anterior descending coronary artery with hemostatic forceps to observe the rats for 20 min and then releasing the hemostatic forceps later for reperfusion. In the control group, no ligation and reperfusion were performed, and the other procedures were the same as the myocardial infarction group. Five rats were randomly executed on Day 14 after the infarction, to detect miR-489 expression after the cardiac muscle cells in the marginal area of the infarction were isolated. All of the procedures above were approved by the Committee of the Third Affiliated Hospital of Qiqihar Medical College.

### 2.3. Cell Culture

Cardiac muscle cells were isolated primarily from cardiac tissues of the control group and tissues from the infarcted margin of the ischemic-reperfusion group. The cardiac tissues were placed into a 5 ml centrifuge tube and cut into pieces, fully blown with 3 ml 0.4% collagen genase and 1.5 ml 0.05% trycrease, and digested at 37°C for 8 min. The mixture was naturally precipitated, the supernatant was discarded, which was finally collected after repeating the above process, at 3000 rpm for 5 min. DMEM containing 10% fetal cow serum was added, and the remaining precipitation was repeated in the digestion steps until the tissue blocks were totally digested. Placing into the incubator for 2 to 3 h, the medium was gently blown after fibroblasts with adherence. All the supernatant was transferred into a centrifuge tube and centrifuged at 3000 RPM for 5 min, with the supernatant discarded, and then cultured in DMEM containing 10% calf serum. Cardiac muscle cells were obtained after fluid exchange 24 h later.

H9C2 cells from embryonic rats' hearts were derived from ATCC, which were placed in a 6-mesh plate (80000 cells/mesh) and cultured in DMEM media with 10% fetal bovine serum and 100 *µ*/m *L* penicillin/streptomycin overnight. Then, the DMEM was replaced with deoxy PBS for 2 h and cultured in the normal environment at 37°C, with 5% CO_2_ and 28% O_2_ for 24 h. Cells without hypoxia/regeneration served as the control group.

### 2.4. Determination of Myocardial Injury Markers (LDH and CK)

48 h after operation, venous blood was taken and LDH and CK in the serum were determined with the corresponding kits, which were purchased from Shanghai Sangon Biotechnology Co., Ltd.

### 2.5. Cell Transfection

Cells with good activity were vaccinated into 6-hole plates and then incubated in 1.5 mL serum-free medium with 500 *μ*L Lipofectamine 3000 (Carlsbad Invitrogen Company, USA) for 24–48 h. Transfected plasmids (miR-489 inhibitor, negative control (NC)) and PI3K/AKT pathway agonist SC79 were provided by GenePharma (Shanghai, China).

miR-489 inhibitor is a specially modified miRNA inhibitor, chemically synthesized. The complementary single chain of chemically modified mature miRNA can inhibit the effects of mature miRNA molecules through specific binding, thus reducing the regulatory effects caused by miRNA in cells.

### 2.6. RNA Extraction and qPCR Amplification

Cells were lysed in 1 mL TRIzol (Invitrogen, Carlsbad, CA, USA) and were fully mixed with chloroform. After centrifuging at 4°C, 12000 rpm for 10 min, the precipitation was incubated with isopropanol and centrifuged again. Finally, the sediment was washed with 75% ethanol, air-dried, and dissolved in water with diethylpyrocarbonate (DEPC). The extracted RNA was reversed on ice to obtain complementary deoxyribonucleic acid (cDNA). The antitranscription template was diluted to a final concentration of 10 ng/*μ*L in DEPC water. qRT-PCR was performed according to the instructions of SYBR Green PCR kit (Takara, Dalian, China), with a total reaction system of 10 *μ*L. qRT-PCR parameters were as follows: predenaturation at 95°C for 15 min, denaturation at 94°C for 15 s, annealing at 55°C for 30 s, and extension at 72°C for 30 s, a total of 40 cycles.

### 2.7. Western Blot

Cell lysate homogenate was extracted after centrifugation for protein supernatant, and protein levels were determined by the BCA method. 20 *μ*g protein supernatant sample was taken for 6% SDS-PAGE. After the gel was removed, it was transferred to the PVDF membrane. The membrane was sealed with 5% skim milk powder at room temperature for 2 h, with anti-Akt, anti-p-Akt, anti-PIP3, anti-Bax, anti-Bcl-2, anti-cytochrome C (Cyt-C), and anti-GSK3*β* antibodies added (diluted at 1 : 1000) and incubated at 4°C overnight. After washing, horseradish peroxide labeled secondary antibody (1 : 1000 dilution) was added and incubated at room temperature for 1 h. The color was developed by chemiluminescence apparatus and analyzed by ImageJ software. Reagents were purchased from AbCAM, Cambridge, MA, USA.

### 2.8. Luciferase Reporter Test

SPIN1 3′UTR containing miR-489 target binding sites of wild-type or mutant sequences were cloned into a carrier of luciferase reporter, which was transfected with miR-489 mimics in H9C2 cells. Then, luciferase activity was determined by a double luciferase reporter analysis system (PROMEGA).

### 2.9. Cell Apoptosis Detection

In the packaged ELISA reaction plate, 20 *μ*L test samples were added to each mesh, 20 *μ*L histone-DNA complex was added as a positive control, 80 *μ*L newly prepared immune reaction mixture (containing anti-histone antibody and anti-DNA antibody) was added to each mesh, oscillated at 300 r/min at the room temperature on the micro-oscillator for 2 h. The liquid in each mesh was poured out. 250 *μ*L incubation buffer was added to wash the samples 3 times, then 100 *μ*L substrate solution (ABTS) was added, and another mesh was added with substrate liquid as a control, which was oscillated at 250 r/min at the room temperature on the micro-oscillator for 5 min, determined by the double-wavelength specific color method (main wavelength, 405 nm; reference wavelength, 490 nm), the value of histone-DNA fragment was expressed as absorbance. The higher the absorbance, the more apoptosis. The test kit was purchased from Roche (Cargo no. 11920685001).

### 2.10. Statistical Analysis

All experiments were independently repeated at least 3 times, with all results represented by mean ± SEM. Data analysis was conducted with SPSS *v* 24.0 software (SPSS, Inc.). Multiple data sets were compared with one-factor ANOVA and Tukey post facto test. Two data sets were compared with unpaired *t*-tests. *P* values were calculated bilaterally, and *P* < 0.05 was defined as statistically significant.

## 3. Results

### 3.1. miR-489 Was Highly Expressed in Cardiac Muscle Cells of Animal Model in the Ischemic-Reperfusion Group

To study the changes of miR-489 during ischemia-reperfusion, the myocardial ischemia-reperfusion model was established in SD rats. Firstly, the levels of serum LDH and CK in the two groups were measured to evaluate whether the establishment was successful. According to the data, there was a significant increase in the levels of LDH and CK of rats in the H/R group compared to the control group (Figure 1(a)). miR-489 expression of cells in the marginal area of myocardial infarction on Day 14 after surgery was determined by qRT-PCR. The results showed that compared with the control group, miR-489 expression in the infarction border zone was increased in the H/R group on Day 14 and Day 28, with a statistically significant difference (*P* < 0.05) (Figure 1(b)).

### 3.2. High Expression of miR-489 in the Animal Model Was Associated with Increased Apoptosis of Cardiac Muscle Cells with Ischemia-Reperfusion

To clarify the relationship between miR-489 expression and the apoptosis of cardiac muscle cells after ischemia-reperfusion, the apoptosis of cells in the infarction border zone was measured by ELISA on Day 14 after operation in both groups. The results showed that increased apoptosis in the H/R group was statistically significant (*P* < 0.05) (Figure 2), so we determined that miR-489 expression was positively associated with the apoptosis of cardiac muscle cells after ischemia-reperfusion.

### 3.3. Inhibition of miR-489 Reduced the Apoptosis of Cardiac Muscle Cells Caused by Ischemia-Reperfusion

To further clarify the effects of miR-489 on the apoptosis of cardiac muscle cells caused by ischemia-reperfusion, H9C2 cells induced by H/R after cell transfection were divided into control group, miR-489 negative control (NC) group, and miR-489 inhibitor group, and miR-489 expression and apoptosis in the three groups were measured, respectively. The results showed significantly decreased apoptosis in the miR-489 inhibitor group compared to that of the control and miR-489 NC groups (*P* < 0.05). See Figure 3.

### 3.4. miR-489 Targeted the Inhibition of SPIN1

It is learned from the Target Scan database query that SPIN1 is the downstream target of microRNA-489. qRT-PCR results showed that SPIN1 expression in H9C2 cells induced by H/R was lower than that in the control group (Figure 4). Double fluorescence reporter enzyme assay validated miR-489 targeting SPIN1 (Figure 4(b)). Thus, we can determine that miR-489 targeted the inhibition of SPIN1.

### 3.5. miR-489 Regulated Cardiac Muscle Cells Apoptosis after Ischemia-Reperfusion by Targeting the SPIN1-Mediated PI3K/AKT Pathway

Previous studies showed that miR-489 plays a biological role in inhibiting PI3K/AKT pathway. In this study, the expression levels of AKT, p-AKT, and PIP3 in three groups of H9C2 cells were determined with Western blot, to clarify the activation of PI3K/AKT pathway. The study showed increased expression levels of p-AKT and PIP3 in miR-489 inhibitor groups compared with those of blank controls and miR-489 NC groups (Figure 5), suggesting that miR-489 may play a biological role in regulating the apoptosis of cardiac muscle cells after ischemia-reperfusion by inhibiting PI3K/AKT pathway.

The expressions of the apoptotic-related proteins (Bax, Bcl-2, Cyt-C, and GSK3*β*) downstream PI3K/AKT pathway in three groups of H9C2 cells were detected by Western blot. The study showed increased Bcl-2 expression and decreased expressions of Bax, Cyt-C, and GSK 3*β* in the miR-489 inhibitor group compared with those in the control and miR-489 NC groups, suggesting that miR-489 can regulate the apoptosis of cardiac muscle cells by inhibiting PI3K/AKT pathway. H9C2 cells were transfected with PI3K/Akt pathway agonist SC79 to detect apoptosis and expressions of apoptotic-related proteins. The results showed decreased apoptosis, increased Bcl-2 expression, and decreased expressions of Bax, Cyt-C, and GSK3*β* in the SC79 group (Figure 5(b)) compared with those of the control and miR-489 NC group (Figure 5(c)). The above results indicate that miR-489 promotes apoptosis via hypoxia/regeneration treatment by inhibiting PI3K/AKT pathway.

## 4. Discussion

With the development of society and economy, as well as people's lifestyle, the impact of risk factors related to cardiovascular diseases on people's health in China seems more significant. It maintains a high incidence of cardiovascular disease, and the coronary artery disease represented by ACS has become one of the major diseases threatening the life and health of people in China. The main pathophysiological mechanism of ACS is acute myocardial ischemia and myocardial injury resulting from internal coronary thrombosis, and maintaining the survival of cardiac muscle cells is of great significance for improving cardiac functions and long-term prognosis in patients with such diseases. In recent years, the extensive use of percutaneous transluminal coronary intervention (PCI) in the acute phase of ACS has significantly reduced mortality in patients. However, during PCI, reperfusion of ischemic cardiac muscle cells may further aggravate cardiac muscle cells injury and even necrosis, commonly known as myocardial ischemia-reperfusion injury (MIRI). MIRI is a complex pathophysiologic process, which is a result of a variety of factors. Studies have shown that the apoptosis, necrosis, and autophagy of cardiac muscle cells caused by important factors, such as oxidative stress, calcium overload, immune response, inflammatory response, and metabolic injury, may be important mechanisms for MIRI [2–4].

Apoptosis is a physiological and pathological process regulated by various genes, including the three pathways of the endoplasmic network pathway, death receptor pathway, and mitochondrial pathway [14]. The pathogenesis and progression of various cardiovascular diseases are associated with close apoptosis and the inhibition or activation of related signaling pathways. Studies have shown that Nrf2/ARE signaling pathway, as an important endogenous antioxidant signaling pathway, plays an antioxidant and cardiac protection role after myocardial ischemia-reperfusion [15–17]. Activation of JAK2/STAT3 pathway has also been shown to reduce MIRI in rats [18–20]. Activation of Wnt/*β*-catenin signaling pathway promotes the apoptosis of cardiac muscle cells by upregulating apoptotic protein Bax and downregulating the expression of antiapoptotic protein Bcl-xl [21]. PI3K/AKT pathway has been proved to be one of the most important signaling pathways in promoting the proliferation of cardiac muscle cells and fighting the apoptosis of cardiac muscle cells [22–24]. PI3K/AKT pathway can play an antiapoptotic role by regulating the activity of Bcl-2 family, which consists of both proapoptotic proteins and antiapoptotic proteins. Bax, as an apoptotic protein, plays a key role in initiating mitochondria-mediated apoptosis [25]. Bcl-2 plays an antiapoptotic role in inhibiting mitochondrial rupture, caspase-3 activation, and Bax cytotoxicity [26, 27]. GSK-3*β* is a key enzyme involved in liver sugar metabolism and can participate in the regulation of apoptosis by affecting the concentration of blood sugar, regulating the proportion of Bax/HKII and mitochondrial permeability, and releasing Cyt-C, as an important component in the respiratory chain involved in redox and energy metabolism and a key substance in the mitochondrial pathway to initiate apoptotic procedures.

Apoptosis plays an important role in MIRI. With the continuous popularization of PCI technology, MIRI has gradually become a prominent problem. Reducing the apoptosis of cardiac muscle cells and increasing surviving cardiac muscle cells after myocardial ischemia-reperfusion is important in improving the prognosis of patients with ACS. In recent years, finding effective means to treat myocardial injury after myocardial ischemia-reperfusion has gradually become a research hotspot. Using antioxidants (hydrogen, NO) [28, 29], calcium overload inhibitors [30], reducing the neutrophils during reperfusion (P selector inhibitors, colchicine, etc.) [31, 32], activating vagus nerve [33, 34], and other methods have been confirmed in some experiments and studies, which can reduce the area of myocardial infarction. However, their roles in reducing the infarction area or improving the prognosis in humans have not been observed. At present, there is no unequivocal and effective clinical treatment method for myocardial ischemia-reperfusion injury. Therefore, it is crucial to explore the factors affecting apoptosis after MIRI and find an effective means to reduce apoptosis after ischemia-reperfusion.

MicroRNA is an endogenous noncoding single-chain small RNA molecule whose main physiological role can be a posttranscriptional regulator of gene expression and play an important role in the occurrence and development of many diseases, especially tumors. In recent years, it has been gradually recognized that microRNA may play a key role in the occurrence and development of MIRI. It has been shown that miR-29a promotes the apoptosis of cardiac muscle cells after ischemia-reperfusion injury by inhibiting IGF-1 [35]. miR-128 can increase the apoptosis of cardiac muscle cells after MIRI by inhibiting PPARG signaling pathway [36]. miR-135a can reduce the apoptosis of cardiac muscle cells in rats after MIRI by targeting regulatory protein tyrosine phosphatase 1B [37]. miR-193b can reduce apoptosis after MIRI in rats, which is a protective factor for MIRI in rats [38]. miR-24-3p, miR-320, miR-298, and miR-140 also play an important role in MIRI [8, 39–41]. Therefore, to explore the role of microRNA in MIRI, we have to find an effective treatment for reducing MIRI. miR-489 is a microRNA associated with malignant tumors found in recent years that can play the role of oncogenes or tumor repressor by regulating the proliferation, differentiation, and apoptosis of human cells. It has been shown that, in ovarian, colon, and glioma cancer, high expression of miR-489 can inhibit the development of tumors by increasing the apoptosis of tumor cells while the loss of miR-489 promotes the development and metastasis of tumors [9–11, 42]. It has also been reported that miR-489 is involved in the inhibition of nerve cell proliferation, induction of apoptosis, and inhibition of neurite growth after spinal cord injury [43]. In recent years, some studies have found that miR-489 plays an important role in the development of myocardial fibrosis (13). However, its effects and specific mechanisms on the apoptosis of cardiac muscle cells after ischemia-reperfusion remains unclear and need to be further discussed.

## 5. Conclusion

In order to investigate the influence of miR-489 on the apoptosis of cardiac muscle cells in MIRI and its specific mechanism, we established a myocardial ischemia-reperfusion model in rats to explore the relationship between miR-489 expression and the apoptosis of cardiac muscle cells after myocardial ischemia-reperfusion. The results showed that the levels of LDH and CK in the serum significantly increased in the H/R group, and miR-489 expression significantly increased in cardiac muscle cells in the infarction border zone, compared with those of the control group. We measured the apoptosis of cardiac muscle cells in both groups, respectively, with ELISA. It increased in the H/R group compared with that in the control group. Therefore, we determined that high expression of miR-489 was associated with increased apoptosis of cardiac muscle cells after ischemia-reperfusion. Subsequently, we knocked down miR-489 expression through cell transection with H9C2 cells induced by H/R to explore the effects of miR-489 expression levels on the apoptosis of cardiac muscle cells due to ischemia-reperfusion. The results showed that the inhibition of miR-489 expression could reduce the apoptosis of H9C2 cells induced by H/R. After querying the TargetScan database, SPIN1 was known to be the downstream target of miR-489. We verified miR-489 targeting SPIN1 through a double fluorescence reporting enzyme test. Previous studies showed that miR-489 promotes apoptosis by inhibiting the SPIN1-mediated PI3K/AKT pathway [9]. To investigate the specific mechanism of miR-489 affecting apoptosis after ischemia-reperfusion, we determined the expressions of PI3K/AKT pathway-related proteins and apoptotic proteins by Western blot and found that H9C2 cells with low expression of miR-489 had increased expressions of p-Akt and PIP3; decreased expressions of proapoptotic genes Bax, Cyt-C, and GSK3*β*; and increased expressions of antiapoptotic gene Bcl-2. The treatment with PI3K/AKT pathway agonist SC79 reduced the apoptosis of cardiac muscle cells after ischemia-reperfusion caused by the high expression of miR-489. We judged that miR-489 can promote the apoptosis of cardiac muscle cells after ischemia-reperfusion by targeting the inhibition of the SPIN1-mediated PI3K/AKT pathway.

In conclusion, our study found that high expression of miR-489 was associated with increased apoptosis of cardiac muscle cells after ischemia-reperfusion, and miR-489 promoted the apoptosis of cardiac muscle cells after ischemia-reperfusion by targeting the inhibition of the SPIN1-mediated PI3K/AKT pathway. Inhibiting miR-489 expression effectively reduced the apoptosis of cardiac muscle cells after ischemia-reperfusion. Therefore, miR-489 is expected to be one of the potential therapeutic targets for reducing the apoptosis of cardiac muscle cells after ischemia-reperfusion.

## Figures and Tables

**Figure 1:** High expression of miR-489 in cardiac muscle cells of animal model in the H/R group. (a) Levels of LDH and CK in the serum in rats of the H/R group increased significantly compared with that of the control group (*n* = 5, *P* < 0.05). (b) miR-489 expression was measured by qRT-PCR after primary separation of cardiac muscle cells in rats. Compared with that of the controls, miR-489 expression was increased in the H/R group on Day 14 and Day 28 (*n* = 5, *P* < 0.05).

**Figure 2:** Increased apoptosis in the myocardial ischemia-reperfusion model. *Note.* Apoptosis of cardiac muscle cells in both groups was measured by ELISA on Day 14 after operation, which increased in the H/R group compared with that of the control group (*n* = 5, *P* < 0.05).

**Figure 3:** Inhibition of miR-489 reduced the apoptosis of cardiac muscle cells caused by ischemia-reperfusion. (a) miR-489 expression in three groups of H9C2 cells was measured by qRT-PCR. (b) Apoptosis in three groups of cells was measured by ELISA. Apoptosis significantly decreased in the miR-489 inhibitor group compared with that of the control and miR-489 NC groups (*P* < 0.05).

**Figure 4:** miR-489 targeted the inhibition of SPIN1. (a) SPIN1 was poorly expressed in H9C2 cells induced by H/R. (b) Dual luciferase report gene analysis confirmed microRNA-489 binding to SPIN1. (c) Matched sequence of SPIN1 and miR-489.

**Figure 5:** miR-489 regulated cardiac muscle cells apoptosis after ischemia-reperfusion by targeting the SPIN1-mediated PI3K/AKT pathway. (a) The expression levels of AKT, p-AKT, and PIP3 in three groups of H9C2 cells were determined by Western blot to clarify the activation of the PI3K/A KT pathway. Increased expression levels of p-AKT and PIP3 in the miR-489 inhibitor group compared with those of the control and miR-489 NC groups suggest that miR-489 may play a biological role in inhibiting PI3K/AKT pathway. (b) H9C2 cells were transfected with PI3K/Akt pathway agonist SC79 to detect their apoptosis. Apoptosis decreased in the miR-489 inhibitor and SC79 groups compared with that of the control and miR-489 NC groups. (c) The expressions of apoptosis-related proteins in the SC79 and other groups were determined. Bcl-2 expression increased and the expressions of Bax, Cyt-C, and GSK3*β* decreased in SC79 and miR-489 inhibitor groups compared to the control and miR-489 NC groups.

## Data Availability

The datasets used and/or analyzed during the present study are available from the corresponding author on reasonable request.
